RETRACTED

# Key Information Extraction of Food Environmental Safety Criminal Judgment Documents Based on Deep Learning

**DOI:** 10.1155/2022/4661166

**Published:** 2022-09-13

**Authors:** Zhijuan Ni

**Affiliations:** School of Political Science and Law, Weifang University, Weifang 261061, China

## Abstract

Food has an impact on everyone's daily life, the long-term stability of the nation, human survival and development, people's lives and health, and the steady advancement of society. A food safety criminal judgment is a legal document used to record the trial of food-related offences. It primarily contains the case's history, information about the parties involved, and the verdict. In order to identify defendants, their charges in court documents, and other important court information, this paper proposes a method for extracting key information from food safety criminal conviction documents based on deep learning. It builds and analyses a hidden Markov model (HMM) based on the corpus of crime-related components, and uses the model trained by a DL neural network to determine the trend of a given data set. In the test result classification task, the results demonstrate that the Transformer model can achieve macro accuracy rates of roughly 0.963, macro recall rates of 0.932, and macro F1 scores of 0.958. Experiments demonstrate the model suggested in this paper's performance and effectiveness in extracting abstract information from food criminal trial documents.

## 1. Introduction

Food security has emerged as one of the most pressing issues facing society today as a result of the growth of the market economy. Food safety issues will be caused by issues with food production and its distribution systems, either directly or indirectly. Judicial documents are authoritative written judgments with force of law rendered by the court acting as the state's advocate on the substantive or procedural issues of particular cases [1]. Criminal judgment records the court's sentencing process, sentencing factors, sentencing justifications, and sentencing outcomes in writing. The defendant's name, the crime's scene, the time it occurred, and the charges are the main pieces of information in the criminal judgment documents published by the court. The focus of this paper is on the uniqueness of text mining in the judicial field as seen in the identification and extraction of defendants and their collecting subjects in criminal judgment documents.

Food safety has evolved into one of the most pressing issues in today's society as a result of the market economy. Food safety issues may arise directly or indirectly as a result of the food production process and its distribution networks. When a court is exercising its judicial authority, judicial documents are authoritative written judgments with a legal effect that are made by the court on behalf of the state regarding the substantive or procedural issues of particular cases. Criminal judgment records the court's sentencing process, sentencing factors, sentencing justifications, and sentencing outcomes in writing. The defendant's name, the crime's scene, the time it happened, and the defendant's criminal conduct are the three main pieces of information in the criminal judgment documents the court issues. The focus of this paper is on the uniqueness of text mining in the judicial field as seen in the identification and extraction of defendants and their collecting subjects in criminal judgment documents. Sichel uses fabricated, specially crafted rules to identify organisational entities [2]. To extract entities, Stahn suggested using a dictionary-based method [3]. To put it simply, it involves creating a domain data set dictionary, and entity extraction is done by comparing the text with related words in the dictionary. The flaw of low accuracy in open tests is evident in Jorge et al's named entity recognition of Twitter text based on a sizable disambiguation corpus. Despite having poor flexibility, texts with fixed formats can still be efficiently and simply written. Not only do we want accurate results, but we also want information about related topics. We can identify text knowledge and mine important information from the text using information extraction technology. We can also determine the relationship between different entities.

RETRACTED

Artificial intelligence researchers have been working on deep learning-based [4] legal text processing technology in recent years in an effort to fully exploit the value of legal text data and lessen the heavy data processing workload of legal professionals. An essential and fundamental task in natural language processing is named entity recognition. The aforementioned situation will not hold if the essential data of the named entities are not extracted. In tasks such as text classification and machine translation, DL has outperformed conventional approaches in terms of natural language processing [5]. This paper uses DL technology to complete the task of tendency analysis of judgment results because this task is comparable to the emotion analysis task in the field of natural language processing. This study establishes the HMM (hidden Markov model) [6] based on the corpus of crime-related components, uses this model to decode and analyse, and then determines the accused entity to carry out the extraction experiment and analyse the results. This study is based on the rule-based extraction and analysis of the time and place of the case with a relatively fixed analysis format.

RETRACTED

### 1.1. Research Innovation

1. The innovation of this paper focuses on solving the problem of entity pair matching in traditional information extraction ideas. Using a one-stage information extraction model based on directed graph structure, the pointing relationship between subject and object can be accurately described.
2. In this paper, the DL-based judgment result tendentiousness analysis model is constructed. By comparing the accuracy of different models in judgment result tendentiousness analysis, the effectiveness of the DL-based model in the judgment result tendentiousness analysis task is verified.

The main body of this paper is divided into five chapters, and its organisational structure and specific content are as follows.

## 2. Related Work

### 2.1. Research Progress of Legal Text Processing

The workload for court staff is rising along with the volume of data. Judges and attorneys should thoroughly research new laws and regulations, as well as those that will be added to or expanded upon existing ones. They should also consult a large number of historical cases as a source of information. The legal text contained in criminal judgment documents, which primarily includes a description of the defendant's information, case, and sentence outcomes, is the most significant data form in the legal field. Legal texts differ from texts in other fields in that they have clear structural elements, strong subject matter, and extensive information. The best legal text technology will significantly enhance the performance of downstream tasks such as modelling, classification, reasoning, and mining.

Zhu et al. put forward a legal text representation model based on the attention mechanism. By training the corpus of judgment documents involving 10 kinds of criminal offences, the latent semantic feature representation vectors based on the facts of the case, the information of the defendant, and relevant criminal law provisions are generated, which greatly improves the performance of the prediction tasks such as crimes, legal provisions and sentences, and the interpretability of the prediction results [7]. Mellish et al. focused their research on how to use the neural network based on attention mechanism to mine cases and describe the logical relationship between different parts, and achieved excellent performance in the task of crime and law prediction [8]. Liu et al. put forward a multichannel attention neural network framework, which only uses three easy-to-obtain labels in training data for supervision to jointly code the case description, defendant information, and legal provisions. The flexible coding method can support different multilabel classification tasks and has achieved good classification performance [9]; Yang et al. put forward a concept of legal dispersion, which measures the similarity of the adjacent node sets of two cases to find a similar case in the citation network [10].

RETRACTED

Tang et al. aiming at the nonaligned bilingual corpus realized the self-expansion method by calculating the local editing distance deviation between the two languages, and realized the named entity recognition under unsupervised learning [11]. Jiang et al. extracted information about specific events from Twitter based on the SVM (support vector machine) model. However, the SVM model is limited to binary judgment, which is not suitable for more complicated named entity recognition [12]. Samawi et al. studied the intelligent proofreading of documents according to the compilation norms of judgment documents, combined with laws and regulations [13]. Wang and Mao proposed to judge the emotional polarity of the whole text according to the correlation between the words and phrases in the text to be tested and the emotional words or phrases in the seed dictionary [14].

### 2.2. Present Situation of DL

DL is not a new method, is originated from the research of artificial neural network, and is a general name for a class of learning methods based on DNN (deep neural network). Subsequently, other depth structure algorithms have been proposed continuously, and important progress has been made in speech, image, and other ability tasks.

With the continuous innovation and development of neural network and DL theory, as well as its mature application in the fields of graphic processing and speech recognition, more and more researchers pay attention to the powerful feature extraction ability and modelling advantages of the DL model. Li and Gong combined the pretrained static word vector and dynamic word vector to represent a piece of text together, and input it into two channels of CNN, which also achieved a good classification effect [15]. Wang and Feng introduced the attention mechanism in the pool layer of CNN (convective neural network) and constructed the middle vector representation of the input text using the long short-term memory, and used it as the attention weight of the text feature vector generated by CNN after convolution and pool. Finally, the text feature vector and attention weight were input into the classifier to complete the classification [16]. Li et al. proposed an RNN (recursive neural network) to predict the tree structure [17].

Guo proposed a scene text segmentation method based on tensor voting [18] to solve the problem that the natural scene text is often polluted by various kinds of noises, such as stripes, highlights, and breaks, which leads to the decline in the accuracy of text recognition. Xu et al. used traditional machine learning methods, including SVM and NB (naive Bayes), to improve the accuracy by combining different classifiers [19]. According to the characteristics of large-scale knowledge base question-answering system, Chen et al. put forward a method of identifying named entities using an alias dictionary combined with an LSTM (long short-term memory) language model, and then disambiguating entities and selecting answers using a two-way LSTM model combined with two different attention mechanisms [20].

RETRACTED

## 3. Methodology

### 3.1. Overall Framework of Key Information Extraction from Food Safety Criminal Judgment Documents

Food safety has become a hot topic when it comes to the safety of human life in today's society because of the rapid advancement of science and technology, which also leads to the constant emergence of new criminal tactics. Such cases are common in judicial practice. These instances of unintentional negligence that result in negative outcomes do not, in accordance with the provisions of criminal law, constitute crimes involving food safety, and they can only be subject to corresponding civil liability and administrative liability. By lowering the constitutive requirements, we can broaden the crime circle and lower the bar for criminal conviction in the area of criminal protection of food safety. The crime of producing and selling food that does not adhere to hygiene standards, as well as the crime of producing and selling toxic and harmful food, shall also carry criminal liability if the behaviour is appropriate unless the makers and distributors of food can demonstrate their lack of malice and implement the necessary measures.

Inconspicuously endangering public health and even posing a threat to lives are harmful substances used in food safety crimes. Its effects cannot be disregarded. The nature of food safety crimes is clear, yet China's criminal justice system is currently unable to effectively reduce violations of food safety. There is still some room for improvement in our legal framework when compared to the food safety legal frameworks of developed Western nations and international organisations. This obviously goes against the goals of democracy and clarity pursued by the legal crime principle, and it also forces judicial staff to constantly switch between criminal law, economic law, and administrative law, decreasing the management effectiveness of judicial organs.

When different scene texts are used, the outcomes will be unsatisfactory if only functions or methods are used. In recent years, research has frequently used hybrid methods or two-layer text location boxes to locate text areas, greatly enhancing the robustness of text location. Text or word recognition is significantly impacted by text distortion, noise pollution, and other factors. Additionally, there are issues that need to be resolved regarding how to extract useful features from text and how to create a suitable classifier. A scene text database with fewer restrictions is necessary to further investigate the primary text extraction technology and perform a thorough performance test comparison.

RETRACTED

According to practical experience, training and forecasting will be very difficult if the named entity recognition model and the relationship classification model are treated as two separate models. We can only use our own synthetic data set for relational classification since our relational classification model is unable to access the real data set. The LSTM network can simultaneously encode information coming from two directions, one of which is front to back, which is how most people read. Reverse, on the other hand, encodes the information in the sentence backwards. Information extraction models based on directed graphs and hierarchical binary labeling models are distinct from one another.

The hierarchical binary labeling model actually decomposes the triple prediction problem into two subproblems:

(1) $$\begin{array}{c} P\left(a,p,o|t\right)=P\left(s|t\right)*P\left(p,o|s,t\right). \end{array}$$

That is, the subject *s* is found according to the text feature *t*, and then the relation *p* and the object *o* are simultaneously searched according to the subject *s* and the text feature *t*. When the feature after the fusion of the subject *s* and the text feature *t* is obtained, this information is meaningfully decoded to obtain the relationship *p* between the object and the corresponding one.

Assuming that a text is segmented and a series of words are *w*_1_, *w*_2_,…, *w*_*n*_, the Skip–Gram model is to seek the parameter *θ* that can maximize the formula:

(2) $$\begin{array}{c} \frac{\arg\max}{\theta }\sum_{\left(c,w\right)\in D}\log\;p\left(c|w,\theta \right), \end{array}$$

where *c* indicates the length of the window; that is, the current word is the center, and there are *c* words before and after it. The larger the value of *c* is, the more comprehensive the semantic relationship between context and context is, and the more accurate the prediction result of the model is, but the higher the training time cost is.

In text classification, according to the number of categories to which document labels belong, it can be divided into single-label (multicategory) classification and multilabel classification. For single-label classification, the existing mature machine-learning and ensemble learning methods can solve this classification task well, and use the Bayesian formula to convert it into posterior probability. If each feature attribute is conditionally independent, the following derivation holds:

(3) Py|xi=Px|yiPyiPx.

RETRACTED

For the same sample, the denominator is fixed, so as long as the numerator is maximized, the decision can be classified according to the posterior probability.

CBOW (continuous bag of words) is a model to predict the occurrence probability of a given word according to its context, assuming a given word sequence (*w*_*t*−2_, *w*_*t*−1_, *w*_*t*_, *w*_*t*+1_, *w*_*t*+2_), where *w*_*t*_ is the word to be predicted at present. The mathematical expression is

(4) $$\begin{array}{c} P\left(S\right)=P\left(w_{1},w_{2},\ldots ,w_{M-1},w_{M}\right),\\ =\prod_{t=1}^{M}P\left(w_{t}|w_{cxt}\right). \end{array}$$

Before the research, we need enough corpus resources as a database, so we first set up a corpus in the field of food safety, preprocess all the corpora in the database, and finally use the processed corpus as a data set for this survey. This document selects 8 types of entities, including time, place, responsible subject, food composition or type, circulation link, cause of the incident, description degree, and countermeasures, and formulates 8 types of corresponding questions. The general information extraction process is shown in Figure 1.

Extraction of the corresponding relationship between the programme state of the parties and the named entity is challenging. On the one hand, the programme state is expressed differently, and on the other hand, the paragraph where the programme state is located contains additional information. Because of this, the extraction process will create unique extraction rules based on the context of features. Following parsing, a candidate is returned, and the candidate text block is then taken into account as a pattern. The text pattern's characteristics are extracted using the proper techniques, and machine learning is then used to categorize and confirm the candidate text regions. Finding entity words and establishing the relationship between the subject and object fall under the purview of the decoder in the two-stage model. The tasks of determining entity words and determining the relationship are carried out by multiple models in the model put forth at this stage.

### 3.2. Implementation of Key Technology of Content Extraction

The only distinction between these regulations and those of criminal law and administrative law is the severity of the behaviour that needs to be modified. A food safety crime is committed if the level of harm caused by the behaviour exceeds the legal threshold. It is necessary to assume the risk of abiding by the criminal law's regulations; if the violation is only general in nature and does not amount to a crime, it shall be specified by administrative law. That is to say, if there is no subjective fault on the part of the offender, no criminal investigation can be conducted. According to the law, behaviour crime and result crime are two types of crimes that put food safety at risk. The basis for the existence of criminal responsibility and the main factor that determines people to bear criminal responsibility for their own actions are typical illegal acts that endanger society and the criminal law. Not all of the issues surrounding the basis of criminal responsibility must be resolved; rather, the rationality of criminal responsibility must be addressed.

RETRACTED

The main goal of data preprocessing is to change the original data's format so that it is compatible with the experimental model. Real-world data frequently contain errors and are lost. In the conventional information extraction model, entities are first identified, and then, the relationships between them are classified. For instance, the subject and object are first located using the entity recognition module, and then, the subject-object pair is entered into the classification model to assess the classification effect. The central step in every classification procedure is feature extraction. The well-designed deep network structure extracts the text features with semantic information and then produces feature vectors that are low in dimension, accurately represent the original text, and suffer from the least amount of information loss.

RNN has unique advantages over variable-length sequence data, so it is widely used in language model training. This document also uses the language model from its training judgment results. In the text vectorization module, we only need to generate a word vector similar to the one-hot representation. This module is divided into three steps: dictionary generation, index mapping, and index sequence generation. To illustrate the overall effect of the DL model, this paper imitates the sentiment analysis model based on dictionary rules and designs a decision result tendency analysis model based on dictionary rules as a benchmark experiment. The model is shown in Figure 2.

Preprocessing the judgment result, creating a trend dictionary, and figuring out the trend based on the dictionary are the three main steps of the model. The trend only needs to compare the text to be tested with the dictionary once the trend dictionary has been generated. The basic concept is to locate a hyperplane that satisfies the classification requirements, and the distance between the training set points and the classification surface is referred to as the classification interval.

RETRACTED

The best classification surface requires that the classification line maximize the classification interval between the two classes in addition to correctly separating the two classes (i.e., the training error rate is 0). Finding frequently occurring itemsets containing litigation state is the behaviour for which the tendency dictionary developed in this paper is a sentence.

In order to generate a tendency dictionary, high-frequency phrases are selected first. In this paper, the Apriori algorithm is used to select high-frequency phrases, and support degree *S* and confidence degree *C* are calculated. According to the given minimum support degree *S*_min_ and confidence degree *C*_min_, the frequent itemsets containing the word *u* are selected. The calculation formula is as follows:

(5) $$\begin{array}{c} \left\{\begin{array}{c} s=\text{count},\\ c=\max\left\{\frac{\text{count}\left(\text{SP}|s\right)}{s},\frac{\text{count}\left(\text{SD}|s\right)}{s}\right\}. \end{array}\right. \end{array}$$

Among them, SP and SD stand for supporting plaintiff and supporting defendant, respectively. The words used in the judgment documents are diversified, such as “defendant, compensation” and “defendant, repayment,” which have the same meaning, but there are different ways of writing them in different judgment documents, which to some extent shows that their terms are not standardized.

The application of HMM in the field of natural language processing usually abstracts the state sequence *S*={*s*_0_, *s*_1_,…, *s*_*T*−1_} corresponding to the observation sequence *O*={*o*_0_, *o*_1_,…, *o*_*T*−1_} into a Markov chain, and models the transition of adjacent state sequences. The formula for calculating the emission probability *b*_*j*_(*k*) of the word *v*_*k*_ under the charge-related component *q*_*j*_ in the emission probability matrix *B* is

(6) $$\begin{array}{c} b_{j}\left(k\right)\approx \frac{C\left(v_{k},q_{j}\right)}{C\left(q_{j}\right)}. \end{array}$$

Among them, *C*(*v*_*k*_, *q*_*j*_) is the frequency of the word *v*_*k*_ with the crime-related component *q*_*j*_ in the corpus, and *C*(*q*_*j*_) is the total frequency of the words with the crime-related component *q*_*j*_ in the corpus.

Transformer proposed a feature extraction mechanism based on attention, which greatly improved the accuracy and efficiency of the model. The core mechanism of the model attention is defined as follows:

(7) $$\begin{array}{c} \text{attention}\left(Q,K,V\right)=\text{soft max}\left(\frac{QK^{T}}{\sqrt{d_{k}}}\right)V, \end{array}$$

where *Q* represents query, which corresponds to the sequence to be expressed; *K*, *V* refer to key and value, corresponding to the sequence used to express *Q*. Softmax is the activation function, which maps the outputs of multiple neurons to the (0,1) interval. Documents are characterized by complex structure and strong contextual relevance. Transformer's attention mechanism can better handle this structure, which requires a large number of contextual text classification tasks.

RETRACTED

Semi-supervised learning does not need a large number of labeled corpora, and the relational extraction model can be obtained by iterative training with a small number of labeled seed samples. Relationship extraction is an important part of information extraction, which is responsible for extracting information from the pairs of entities in the text, and identifying the relationship types between entities through a semantic understanding of the text context. The evidence item relation extraction model proposed in this paper transforms the text into a word vector containing contextual semantic information. Then, the text features are processed by CNN to obtain local features. Finally, the Softmax classifier is used to classify relations, and the model structure is shown in Figure 3.

In this paper, two CNN convolution models with convolution kernel steps of 2 and 3 are built, respectively, which are used to extract the text information of legal decisions between 2 and 3 words. The convolution operation contains a convolution kernel *w* ∈ *R*^*h*×*h*^, and the filter is applied to the window of the *h* word to produce a new feature. The formula is

(8) $$\begin{array}{c} c_{i}=f\left(w\cdot x_{i:i+h-1}+b\right), \end{array}$$

where *b* is an offset term; *f* is a nonlinear function; and “·” means dot multiplication between matrices.

In the output layer of the entity relationship extraction model, the output vector of each output node is converted into probability by the Softmax layer, and the word corresponding to the output node with the highest probability is found as the relative word of prayer. The formula for probability conversion of related words is as follows:

(9) $$\begin{array}{c} P\left(q|S\right)=\text{Soft Max}\left(w_{v}V+b_{v}\right), \end{array}$$

where *P*(*q|S*) is the probability value of the relative word; *S* is the input sentence; *q* is the relative word of prediction; *w*_*v*_ is the weight; *V* is the output vector; and *b*_*v*_ is the offset vector.

RETRACTED

The endpoint model based on the self-attention mechanism is the work of scope extraction using the self-attention mechanism. Its core lies in compressing the feature *X*_*i*_ to a numerical value using FCN (fully connected neural network) layer with shared parameters, and then carrying out weighting operation. Its formula is as follows:

(10) $$\begin{array}{c} Y=\sum_{1}^{n}a_{i}*X_{i}. \end{array}$$

Compared with the first two subsection models, the self-attention-range extraction model can encode the middle words of entity words, and a group of FCN models are set up to compress and reduce the data dimensions.

## 4. Experiment and Results

This experiment is based on Python language, using TensorFlow and PyTorch frameworks to build the DL model, and the MySQL database to store and call data. The data set of this experiment is divided into 4 : 1, and there are nearly 5,000 valid sentences in the training set. It is necessary to set the word embedding layer to use 100-dimensional GloVe (Global Vectors for word representation), and the neural network output vector dimension is 128 dimensions. In order to show the effect of double networks and their attention models, a series of comparative experiments were conducted on the same data set using the traditional neural network model and this model. The specific experimental results are shown in Table 1.

As can be seen from Table 1, the accuracy, recall, and F1 value of this model on the experimental data set are 0.901, 0.881, and 0.895 respectively, and the overall performance is better than that of CNN and RNN models. Among them, “full-text extraction” and “database extraction” are candidate response sentence extraction strategies. One is to take all the sentences in the candidate documents as candidate response sentences, and the other is to extract the candidate response sentences using the food safety incident database. For relation extraction, the dual network model used in this paper has better feedback on sentence structure and will not discard more useful information brought by vertical domain vocabulary.

Taking consumer food safety as an important standard of food evaluation, the proliferation of inferior food in China's market is not conducive to protecting consumers' health, safeguarding consumers' legitimate rights and interests, and safeguarding the legitimate operation of regular food enterprises. On the one hand, it greatly reduces the possibility of people committing other crimes that threaten food safety in China, and can play a special role in risk prevention and control; on the other hand, the punishment of crimes endangers food safety. In order to improve the main sanction types of food safety crimes in China, it is in line with the complex and diverse crime characteristics of food safety crimes in China.

RETRACTED

HMM and NB, which have been trained by corpus, are used to mark crime-related components of different sizes, extract summary information from criminal conviction files, and compare the accuracy and recall performance of the algorithms under different corpus sizes, as shown in Figure 4.

It can be found that, on the whole, the accuracy and recall of HMM are higher than those of NB, and with the increase in training sets, the gap between the two gradually widens. This is because NB assumes that every word in the word sequence is independent of each other, and the words at any given time only depend on the marking state at that time. Therefore, compared with HMM, NB's disadvantages in accuracy and recall are highlighted by the increase in the corpus of crime-related components used for training.

With the continuous expansion of case files, case-like retrieval is of great significance to improve the work efficiency of legal practitioners, and high-quality case-like submission results will also help Chinese laws to be closer to the goal of “case-like” files. Sentences of the first instance and the second instance can be distinguished directly by the name of the sentence, and then part of the sentence can be cut by the fixed template of civil sentences of the first instance and the second instance as shown in Table 2.

Using the standard model framework and model parameters, the performance of the Transformer model on the civil case sentence classification data set is always better than all three models of RNN, CNN, and LSTM. In the first-level judgment result classification task, the accuracy rate can reach about 0.963, the Recall rate can reach 0.932 and the F1 can reach 0.958. In order to explore the influence of neural network layers on the task of trend analysis of decision results, based on the LSTM model, this paper uses 1-layer LSTM to 20-layer LSTM for comparison.  Figure 5 shows the experimental results of neural networks from different depths on the complete data set.

It can be seen that properly increasing the number of neural network layers can improve the accuracy of decision-making result tendency analysis, but it will decrease after increasing to a certain extent, which is mainly because the model is overfitted during training, which leads to the decrease in prediction accuracy. Therefore, the number of DL network layers is not as high as possible. According to the above experimental results and analysis of results, in industrial production, if DL-based models are used to deal with decision-oriented tasks, attention should also be paid to the accuracy of the models, and an appropriate number of neurons should be selected during training. In order to better present the experimental results, in this paper, in the comparison between the model and LSTM, we list the experimental results in the data set in the form of Figures 6 and 7. Data sets are presented in different ways, and experimental analysis is based on all data sets, which will be described in detail in the analysis section below.

RETRACTED

Despite the fact that words within a given dimension are not fixed, the 50-dimensional word vector representation of various words is effective at differentiating between them. The sliding window's size can be adjusted, allowing for the local learning of the information that lies between words and the effective suppression of noise. The difference in feature vector representation between samples, particularly when the sample data are unbalanced, is incredibly small. Because samples with many categories will significantly interfere with samples with few categories, labels with high frequency will be more likely to be correctly predicted. Although it increases the variance in input characteristics between documents, it still only includes data on the frequency of words in documents and not any other information about the semantic structure of documents.

This article set up 100 training sessions, because the accuracy, recall, and F1 value are all indicators to judge whether a model is good or bad, but F1 value is the harmonious average of accuracy and recall. When it is very high, the F1 value will be very high, so F1 value is selected as the model detection mark in model training. The F1 value trend of the training model in this document is shown in Figure 8.

As can be seen from Figure 8, the model added with the attention mechanism in this document is a better model for the identification of people, time, place, and other named entities in the field of food safety. A high-precision named entity recognition model is the key to ensure the smooth development of the preliminary work, whether in the field of food safety research or in the construction of question-answering system and related knowledge map. Considering the public interest of food safety, legislators have adopted a zero-tolerance attitude towards food safety crimes. The application of the strict responsibility system is strictly limited, and the applicable areas are those crimes that violate the indefinite majority and cause damage or threat to public security, which may constitute intentional or negligent crimes. In terms of legislation, China's food safety criminal law can be more perfect, and in practice, it can improve the efficiency of handling cases, realize the shock of food safety crimes, and meet the practical needs of intensifying the crackdown on food safety crimes.

RETRACTED

## 5. Conclusions

The entities in food safety incidents not only have multidimensional semantic knowledge but also are important knowledge units that constitute food safety incident response strategies. Based on the study of corpus, DL obtains the parameters of the HMM model and carries out the summary information of judicial texts, especially the identification and extraction of defendants and their collecting subjects. Using the standard model framework and model parameters, the Transformer model can achieve macro accuracy rate of about 0.963, macro recall rate of 0.932, and macro F1 score of 0.958 in the classification task. The experimental results show that the method described in this paper is effective and can achieve the extraction purpose with a better performance index.

## Figures and Tables

**Figure 1:** Key information extraction process.

**Figure 2:** Analysis model of judgment result tendency based on dictionary rules.

**Figure 3:** Evidence correlation extraction model.

**Figure 4:** Curve of accuracy and recall rate of summary information extraction.

**Figure 5:** Comparison of neural networks in different depths.

**Figure 6:** Performance of this model.

**Figure 7:** LSTM model.

**Figure 8:** Model training F1 value trend.

**Table 1:** Performance comparison of different models.

Model	Accuracy	Recall	*F*1 value
Model of this paper	0.901	0.881	0.895
RNN	0.635	0.068	0.674
CNN	0.759	0.726	0.735
LSTM	0.089	0.863	0.801

**Table 2:** Model index comparison.

Model	Macro accuracy	Macro recall rate	Macro *F*1 value
Transformer	0.963	0.932	0.958
RNN	0.921	0.933	0.908
CNN	0.936	0.921	0.916
LSTM	0.909	0.903	0.922

## Data Availability

The data used to support the findings of this study are available from the corresponding author upon request.
